# Deficient for endoplasmic reticulum calcium sensors Stim1 and Stim2 affects aberrant antibody affinity maturation in B cells

**DOI:** 10.18632/oncotarget.11659

**Published:** 2016-08-27

**Authors:** Xuhua Mao, Jianfeng Zhang, Yue Han, Chao Luan, Yu Hu, Zhimin Hao, Min Chen

**Affiliations:** ^1^ Department of Clinical Laboratory, Yixing People's Hospital, China; ^2^ Department of Preventive Health Care, the Second Affiliated Hospital of Southeast University, China; ^3^ Jiangsu Key Laboratory of Molecular Biology for Skin Diseases and STIs, Institute of Dermatology, Chinese Academy of Medical Sciences, China

**Keywords:** B cells, calcium influx, Stim1, Stim2, antibody affinity, Immunology and Microbiology Section, Immune response, Immunity

## Abstract

Antigen specific B cells undergo a process termed affinity maturation in the germinal centers of secondary lymphoid organs where B cells with high affinity receptors are selected to mature into antibody-producing cells or to the memory B cell pool. It is known that B cell antigen receptor (BCR) signaling plays pivotal role in this selection process. Calcium influx is an essential component of BCR signaling. The current report is to determine the effect of calcium influx on antibody affinity maturation. In our studies, mice deficient for both endoplasmic reticulum calciumsensor Stim1 and Stim2 was immunized with T-cell dependent and independent antigens. Antibody affinity was measured by ELISA. We demonstrated that Stim1 &Stim2 deficient B cells exhibit accelerated pace of affinity maturation compared to wild type controls while the overall antibody production was not dramatically impaired to T-independent antigen immunization. In conclusion, calcium influx plays an important role in antibody affinity maturation in humoral immune responses. The knowledge can be used in manipulate humoral immune response for the design of effective vaccines.

## INTRODUCTION

Calcium influx plays pivotal role in signaling downstream of immune receptors including B and T lymphocyte antigen receptors (BCR and TCR). Upon engagement with cognate antigens, BCR or TCR activates phospholipase C, which in turn hydrolyzes phosphatidylinositol 4,5 biphophate (PIP2) into inositol 1,4,5-triphohphate (IP3) and diacylglycerol. IP3 binds to IP3 receptors in the endoplasmic reticulum (ER) membrane and activates Ca2+ release from ER lumen. Recent studies have elucidated that calcium release from ER activates specific channels on the plasma membrane called Calcium-Release Activate Calcium Channels (CRAC channels) [1]. CRAC channels consist of ER sensors namely Stim1 and Stim2 as well as the plasma membrane pore-forming unit Orai. Upon the depletion of calcium from ER lumen, ER resident proteins Stim1 and Stim2 forms multimers that translocate to the sites of ER-plasma membrane apposition, where Stim proteins mediate the opening of Orai channels on plasma membrane that in turn mediate calcium influx into cytoplasm [1]. The pivotal role of calcium signaling in immune cells has been well studied in the past few years. Calcium influx is essential for mast cell degranulation and lytic function of cytotoxic T cells. Sustained calcium influx is indispensible for antigen receptor induced cell proliferation and cytokine production by T cells, B cells, NK cells and mast cells [2]. In T cells, calcium signaling is especially important for the development and function of T regulatory cells, therefore, T cell specific deletion of Stim genes led to malfunction of T regulatory cells (Tregs) and autoimmunity [3]. All these functions of calcium signaling in immune cells can be traced back to the activity of transcription factor-nuclear factor of activated T cells (NFAT) [4, 5]. NFAT is constitutively phosphorylated and sequestered in the cytoplasm. Calcium influx activates the calmodulin (CaM)-dependent phosphatase calcineurin that dephosphorylates and activates NFAT. Dephosphorylated NFAT then translocates to the nucleus and activate gene transcription.

B cells are essential for humoral immune response. Engagement of BCR on B cell surfaces stimulates the activation of B cells into antibody-secreting plasma cells that constitute the first wave of IgM antibodies after immunization [6–8]. However, production of high affinity antibodies to T cell dependent antigens relies on antigen-specific B cells to enter a specialized histological structure in the follicules in secondary lymphoid organs, namely the germinal centers (GC). In GCs, B cells proliferate and undergo somatic hypermutation (SHM) of the immunoglobulin variable region and class switch. Since these SHM are random, high affinity antibody-producing cells are selected at the cost of apoptosis of B cells with low affinity to cognate antigens [9–11]. Over the past decade, much has been known about how B cells undergo somatic hypermutation and selection. Specifically, signaling strength downstream of BCR plays an important role in the process of selection of high affinity antibody producing B cells. Whereas B cells with high affinity BCRs are presumably selected for the higher binding avidity to the cognate antigens presented on follicular dendritic cells (FDCs), those with lower affinity, or with irrelevant antigen specificity or self reactive BCRs are eliminated or not selected for subsequent proliferation owing to lower BCR signaling strength [12–14].

Calcium signaling plays an important role in B cell-mediated immune response [1]. It has been reported that calcium signaling is indispensable for the specific regulatory B cell type B10 B cell development and therefore contributes to inhibition of autoimmune diseases such as that in the mouse model of multiple sclerosis (MS) [15]. However, it is not clear how calcium signaling affect germinal center reaction and antibody affinity maturation. We report here that despite of the fact that B cell intrinsically deficient for both Stim1 and Stim2 proteins are unable to proliferate in response to BCR crosslinking, mice with B cell specific deletion of both Stim proteins were able to mount effective humoral immune response to both T-independent (TI) and T-dependent (TD) antigens. However, antibody affinity in STromal Interacting Molecule (Stim) deficient mice matured at an accelerated pace in comparison to that in wild type control mice. These observations provided the basis for enhancing humoral immune response to achieve high titer antibodies by manipulating calcium signaling in B cells.

## RESULTS

### Simultaneous deficiency of both Stim1 and Stim2 in B cells does not impair B cell development

Mice carrying LoxP flanked Stim1 and Stim2 gene (floxed [f]) were crossed with mb-1 Cre mice which carries a Cre gene knocked into the Mb1 locus to generate Stim1 f/f, Stim2 f/f, mb1Cre+ mice and Stim1f/+, Stim2 f/+, mb1Cre+ mice were used as wild type control. Mb1Cre mediates recombination at the early stage of B lymphopoiesis [16]. Different compartment of B cells including that in spleen, bone marrow and peritoneal cavity were analyzed for developmental defect in the absence of Stim proteins. Flow cytometry analysis of B cells in the bone marrow, spleen and peritoneal cavity have shown that pre- and pro-B cells as well as immature and mature circulating B cells in the bone marrow from Stim1&2 f/f, mb1Cre+ mice are similar to that in Stim1f/+, Stim2 f/+, mb1Cre+ mice. Similarly, marginal zone B cells, immature and mature follicular B cells in the spleen, as well as B1a and B1b B cells in the peritoneal cavity were not affected by the ablation of expression of Stim proteins (Figure 1A-1C). Consistent with previous report [15], those results indicated that Store Operated Calcium influx is not essential for B cell development.

**Figure 1:** Simultaneous B Cell Specific Deletion of Stim1 and Stim2 Does Not Affect B cell Development **A.** Representative FACS panel showing the percentile of B220 and CD117 positive pro B cells; B220+, CD25+ Pre-B cells; the B220+, IgMhi recirculating B cells and the B220 intermediate, IgM bright immature B cells in the bone marrow from the control Stim1f/+, Stim2 f/+, mb1Cre+ and the DKO Stim1 f/Δ, Stim2 f/f, mb1Cre+ mice. **B.** Representative FACS panel showing the B220 positive AA4.1 negative immature B cells and B220 positive, AA4.1 positive mature B cells; the transitional T1, T2, T3 B cells as well as the CD23 dull, IgM positive marginal zone (MZ) Bells and CD23 bright, IgM positive mature B cells in the spleen of control and Stim 1&2 DKO mice. **C.** B1 B cells in the peritoneal cavity and germinal center B cells in Peyer's patch from control and Stim 1&2 DKO mice. **D.** Absolute number of pro-B, pre-B, immature B and recirculating B cells in the bone marrow of control and Stim1&2 DKO mice. **E.** Percentile of Total B cells, Immature B cells, marginal zone (MZ) B cells and follicular (FO) B cells in the spleen of control and Stim1&2 DKO mice.

### Stim1 and Stim2 are redundant for BCR-crosslinking-induced calcium influx, but Stim1 is essential for sustained calcium influx in B cells

To explore the role of Stim1 and Stim2 in BCR-induced calcium influx in B cells, we purified total B cells from spleen of wild type control and Stim1&2 DKO mice by CD43 magnetic beads depletion. Anti-IgM F(ab)2 crosslinking-induced calcium influx is dramatically reduced in Stim1&2 DKO B cells in comparison to the wild type control B cells (Figure 2A). When ionomycin was added into the culture, calcium influx was massively increased in wild type cells, however, no such effect was observed in Stim1&2 DKO B cells (Figure 2A). These results indicated that Stim1 and stim 2 are essential store calcium depletion sensor for BCR-induced calcium influx in B cells. To further investigate the impact of Stim protein deficiency on BCR-induced calcium influx in sub-populations of B lymphocytes, total spleenocytes were pre-labelled with anti-AA4.1, B220, CD23 and IgM fluorescent antibody, then loaded with Indo-I. Different populations of B cell subsets were gated based on cell surface staining and calcium influx was measured by flow cytometry. While wild type B cells presented a sustained calcium influx upon anti-IgM (Fab)2 stimulation for the 300 seconds time window of analysis, this effect was completely abrogated in Stim1&2 DKO immature (B220+, AA4.1+) and follicular (B220+, AA4.1-, CD23hi IgMhi) B cells. Whereas, Stim 2 deficient Immature and Follicular B cells showed similar calcium influx in comparison to their wild type counter parts, the same subsets of B cells displayed defect in sustained calcium influx in the absence of Stim1. These observations suggest that although Stim1 and Stim2 are redundant for the initial calcium influx induced by BCR cross-linking in immature and follicular B cells, sustained calcium influx depends on Stim1 in these cells. Interestingly, in Marginal Zone (B220+, AA4.1-, IgMhi, CD23 intermediate) B cells, BCR-crosslinking induced calcium influx is not affected by single deficiency of Stim1 or Stim 2, suggesting Stim proteins are redundant for IgM cross-linking induced calcium influx in this subset of B cells. Although calcium influx was dramatically decreased in Stim1&2 DKO marginal zone B cells, it was not completely abrogated as observed in immature and follicular B cells, indicating that other calcium channels may function in marginal zone B cells in addition to store-operated calcium pathways.

**Figure 2:** Compromised calcium influx induced by BCR crosslinking in Stim1&2 DKO B cells **A.** Calcium mobilization monitored by Indo-1 AM imaging. B cells purified from spleen were stimulated with 10μg/ml anti-IgM F(ab)2 for 300 seconds followed by 500nM Ionomycin. **B.** Gating strategy for immature B cells, marginal zone B cells and mature follicular B cells for calcium influx monitoring on FACS depicted in Fig.2 **C. D. E.** Calcium influx in immature B cells (C); mature follicular B cells (D) and marginal zone B cells (E) in spleen from mbCre+ control, Stim1 f/f, mb1Cre+, Stim2 f/f, mb1Cre+ and Stim1&2 f/f, mb1Cre+ (DKO) mice.

### Defective BCR-crosslinking-induced proliferation but intact immunoglobulin isotype switch in Stim 1&2 DKO B cells

To further investigate the impact of Stim deficiency on B cell function, na.ve B cells were purified from total spleenocytes by CD43 depletion and labeled with CFSE. These cells were then stimulated with different combination of stimulants to induce Immunoglobulin class-switch reactions. Cell proliferation was determined by flow cytometry analysis in combination with immunoglobulin subclass cell surface staining. While both wild type and Stim1&2 DKO cells showed similar proliferation profile in response to TLR9 ligand CpG and TLR4 ligand LPS, Stim deficient B cells failed to proliferate in response to BCR crosslinking (Figure 3A). When naïve B cells were stimulated with LPS in the presence or absence of IL-4, γ-interferon, TGFβ, the number of B cells switched to IgG3 (LPS only) or IgG1 (LPS+IL-4), IgG2 and IgA were similar between wild type and the Stim deficient B cells, suggesting Store-Operated Calcium (SOC) channel is not important for immunoglobulin class switch. Accordingly, when immunoglobulin subclasses in the serum from mice without immunization were measured, the level of all immunoglobulin subclasses were not altered dramatically in the absence of Stim proteins in B cells (Figure 3B & 3C).

**Figure 3:** Impaired proliferation upon BCR crosslinking in Stim1&2 DKO B cells **A.** Proliferation of control or Stim1&2 DKO B cells stimulated with TLR9 ligand CpG, TLR4 ligand LPS and anti-IgM F(ab)2 for 72 hours. **B.** Class switch in control and Stim1&2 DKO B cells stimulated with LPS or LPS + IL-4 into IgG3 and IgG1. **C.** Serum level of immunoglobulins IgM, IgG1, IgG2a, IgG2b, IgG3 and IgA in control mb1Cre+, Stim1&2 DKO and Stim2 f/f (control as well) mice.

### Aberrant afinity maturation in Stim-deficient B cells

The failure of Stim deficient B cells to proliferate in response to BCR crosslinking *in vitro* prompted us to reason that these B cells may be incapable of raising an effective humoral immune response. However, as reported before [15], when immunized with alum precipitated T cell independent antigen 3-hydroxy-4-nitro-phenylacetyle coupled to Ficoll (NP-Ficoll) or T cell dependent antigen 4-hydroxy-3-nitrophenylacetyl chicken γ-globulin (NP-CGG), total NP-specific IgM, IgG3 or IgG1 antibody titers are similar between the wild type control and the Stim DKO mice (Figure 4A & 4B). Consistent with previous report, and for reasons, yet, unclear to us, Stim molecules are not essential for antibody-producing humoral immune response. To further characterize the humoral immune response to TD antigens, we measured affinity maturation of NP-specific serum Igs after immunization with100μg of alum precipitated NP-CGG using differential ELISA. The differential ELISA methods use different ratio between hapten (NP) to protein (BSA) conjugate as coating antigen to measure high affinity (i.e. antibodies binding to low NP number BSA (NP6-BSA) and total antibody (i.e. antibodies binding to high NP number BSA (NP30-BSA)). When immunized with T-cell dependent antigen NP-CGG precipitated with Alum, the high affinity anti-NP IgG1 antibody titer (measured by using low density NP6-BSA) are significantly higher in Stim DKO mice in comparison to wild type control mice (Figure 4C). This is an indication that antibody affinity is maturing in a faster pace in the absence of Stim proteins in B cells. When we checked the number of germinal center B cells, the number is not significantly increased in Stim DKO mice in comparison to that from wild control mice (data not shown). It is known that in C57BL/6 mice, the V186.2 VH gene primarily joined to the D segment DH16.1 and JH2 J segment dominates the primary anti-NP responses and there is peculiar pattern of somatic hypermutation for generating high affinity IgG1 (γ1λ1) NP specific antibodies in which high affinity anti-NP antibodies acquire a tryptophan to leucine mutation at position 33 (W33L) [17, 18]. B220+, CD38intermediate and CD95hi germinal center B cells from spleens of mice 7 days post-immunization with NP-CGG were sorted out. Rearranged VH186.2-DH16.1-JH2 gene segments were sequenced,. As shown in Figure 4E, there is a higher frequency of mutations rates in Stim DKO germinal center B cells in comparison to that from C57BL6 wild type control B cells. More importantly, the W33 to L mutation rate is much higher in Stim DKO germinal center B cells than the wild control B cells. These results are consistent with the increased affinity maturation of the serum IgG1 against NP haptens as measured by differential ELISA (Figure 4C).

**Figure 4:** Aberrant affinity maturation in Stim1&2 DKO B cells **A.** anti-NP (Nitrophenyl) specific high affinity antibody titer (measured by NP6-BSA ELISA) and total anti-NP specific IgG1 antibody (measured by NP30-BSA ELISA) from mice immunized with NP-CGG on Day 7 and Day 14. **B.** The ratio between high affinity and total NP-specific IgG1 antibody in mice immunized with NP-CGG in alum on day 7 and day 14. **C.** Gating strategy for sorting of germinal center B cells on Day 7 after NPCGG immunization. **D.** Summary of sequencing result of VH186.2-JH2 Gene segment in GC B cells from control or Stim1&2 DKO mice. (a: mutation frequency of all mutations, b: frequency of the W33L specific mutations).

## DISSCUSION

To study the function of calcium sensors Stim1 and Stim2 in controlling B cell immune response, we have generated B cell-specific deletion of Stim1 and Stim2 in mice. Consistent with previous findings [15], our results showed that Stim1 and Stim2 are not required for B cell development, antibody production upon immunization and antibody class-switches. However, B cell antigen receptor (BCR) induced calcium influx and B cell proliferation is profoundly defective in these B cells. A closer look at calcium influx in different subsets of B cells as well as B cells at different developmental stages, we found that Stim1 and Stim2 functions differentially in mediating calcium influx. In immature and follicular B cells, Stim1 and Stim2 are redundant in mediating the initial calcium influx. However, Stim1 plays a more important role in maintaining the sustained calcium influx in these B cells. In contrast, in marginal zone B cells, either Stim1 or Stim2 is sufficient to support the initial and the sustained calcium influx induced by BCR. More importantly, there seemed to be another molecular mechanism that mediates BCR-induced calcium influx in marginal zone B cells that is independent of Stim1 or Stim2. This Stim1&2 independent calcium influx, although lower than wild type B cells, is still substantial.

Despite of the profound defect in BCR-induced calcium influx and proliferation, Stim1 and Stim2 deficient mice were able to mount robust humoral immune response against both TI and TD antigens. Furthermore, our data also indicated that in the absence of Stim1 and Stim2, the antibody affinity maturation is accelerated. Consistently, we found that at the molecular level, Stim1 and Stim2 deficient germinal center B cells displayed higher frequency of somatic mutations. More importantly, the selection for W33L upon NP-CGG immunization is also dramatically enhanced. These observations suggested that Stim proteins play an important role in antibody affinity maturation. Antigen specific B cells that enter the GC undergo proliferation and somatic hypermutation (SHM) in the dark zone. These B cells then enter the light zone of GC and interact with cognate antigens from follicular dendritic cells and processing and presenting these antigens to follicular T help cells. The competition between B cells for Tfh cells dictates that only high affinity antibody producing B cells were selected, while these B cells with lower affinity either undergo apoptosis or go back into the dark zone for another round of hypermutation and selection [19–21]. The higher frequency of mutations in Stim deficient B cells in comparison to wild type control B cells suggested that Stim protein-mediated calcium signaling downstream of BCR are important for the upregulation of components of the SHM machinery and therefore increased the efficiency of SHM. In addition to the SHM machinery, cytokines also plays important role in SHM and the selection for high affinity antibody-producing GC B cells. Among these cytokines, IL-10 has recently being shown to be an important GC reaction regulator [22]. IL-10 from follicular T regulatory cells (Tfr) can directly act on Tfh cells, inhibiting Tfh cells function and therefore negatively affect GC reactions and antibody affinity maturation [15,23]. It is interesting that Matsumoto, et al recently reported that Stim1&2 plays an essential role in BCRinduced IL-10 production in B cells activated by BCR crosslinking and this defect led to exacerbation of experimental autoimmune encephalomyelitis in a mouse model of multiple sclerosis. One possible explanation of our results is that the B-cell originated IL-10 may also directly act on Tfh cells in a paracrine manner to inhibit GC reactions as a feedback mechanism. In the absence of Stim proteins, BCR-induced B cell production of IL-10 is severely impaired and therefore there is exacerbated GC reaction, which in turn leads to higher SHM and increased pace of affinity maturation.

In conclusion, antibody immune response remains to be the fundamental mechanism for vaccination mediated protection against infectious pathogens. Our studies elucidated a mechanism that has not been reported before that by manipulating calcium signaling in B cells may increase the affinity maturation and therefore provided the basis for developing more effective designs for novel vaccines to benefit the human heath welfare.

## MATERIALS AND METHODS

### Mouse strains

The Stim1fl/fl and Stim2fl/fl mouse strains were purchased from Jackson Laboratory (Stock NO: 023350 for Stim1 and 026638 for Stim2). Mice carrying these conditional alleles were crossed with mb1-knockin cre mice [16] to generate a compound transgenic mouse strain. Mice were kept in SPF facilities and all mouse protocols were approved by the Institutional Animal Care and Use Committee.

### Flow cytometry

Single-cell suspensions prepared from various lymphoid organs were stained with the following monoclonal antibodies conjugated to phecoerythrin (PE), Peridin-Chlorophyll (PerCP), allophycocyanin (APC), or biotin: anti-CD19, Fas (anti-CD95), B220/CD45R (clone RA3-6B2) (all from BD Pharmingen), and anti-CD38 (clone 90, eBioscience). All samples were acquired on a FACSCalibur (BD Biosciences, San Jose, CA) and results were analyzed with FlowJo (Tree Star, Ashland, OR) software. Germinal Center B cells (B220+, CD38lo Fashi) and non-GC (B220+CD38hiFas-) were sorted on FACSAria (BD), using the DIVA version 5.0 software.

### Immunization and ELISA

Mice were immunized with 100μg of T-dependent (TD) antigen NP-CGG (4-hydroxy-3-

nitrophenylacetyl chicken γ-globulin, Biosearch Technologies, Novato, CA) or T-independent antigen NP-Ficoll (Biosearch Technologies) in Imject Alum (Pierce Biotechnology, Rockford, IL) intreaperitoneally. Before and on day 7, 14, 21 post immunization, mice were bled or sacrificed for analysis. Serum samples were analyzed by ELISA with coating and detection antibody purchased from Southern Biotech (Birmingham, AL) or Biosearch Technologies.

### *In vitro* B lymphocyte activation, proliferation and class switch assay

B lymphocytes were purified by CD43 depletion using anti-CD43 magnetic beads (Miltenyi Biotech). B cells were activated *in vitro* at a density of 5×105 cells /ml either with 20μg/ml of LPS, 2μg/ml anti-CD40 (1C10, eBioscience) or 10μg/ml of goat anti-mouse IgM, μ-chain specific F(ab′)2 fragment (Jackson Immunoresearch, West Grove, PA) in Dulbecco's modified Eagle's medium (DMEM) supplemented with 10% feta calf serum, L-glutamine, penicillin-streptomycin, nonessential amino acids, sodium pyruvate, HEPES and 2-mercaptoethanol (Invitrogen). For proliferation assay, CD43 depletion purified B cells were labeled with 1nM CFSE for 10 min at 37°C in 5%CO2, followed by 2 wishes with cultural medium. Labeled cells were then activated as described above for 3 days. Proliferation was monitored by FACSCalibur, and data were analyzed using FlowJo software. For immunoglobulin class switch assay, purified B cells were labeled with CFSE and activated by LPS in the presence of IL-4 (IgG1), γ-interferon (IgG2a,b), TGFβ (IgA). On day 4, cells were stained with antibodies again each individual Ig isotype specific antibody and analyzed by FACSCalibur.

### Single cell [Ca2+]i imaging

This was done precisely as described in Oh-hora, et al [3], except for B cells. Briefly, splenic B cells purified by CD43 depletion were cultured overnight RPMI 1640 with 10% FBS for 16 hours followed by loading with calcium indicator Fura-2-AM (1μM, Invitrogen) at a density of 1×106 cells/ml for 30 min at 22-25°C. Cells were then attached to poly-L-lysine-coated coverslips for 15 minutes. B cells were then stimulated with anti-IgM F(ab′)2 fragment by perfusion of cells with the antibody at 10μg/ml. For long term Ca2+ imaging, Fura-2-AM labeled B cells were stimulated with 10nM PMA and 0.5μM ionomycin in Ringer's solution containing 2mM Ca2+ supplemented with 2% FBS. During image acquisition, cell was constantly perfused with buffer warmed up to 37°C. [Ca2+]i was measured and analyzed as described [24]. Ca2+ influx rates were inferred from the maximum rate of the initial increase in [Ca2+] in 0.2-2mM extracellular Ca2+ expressed at the ration ‘Δ[Ca2+]i/Δt’, where ‘Δ[Ca2+]i’ is the maximum difference in [Ca2+]i over a 20 second time interval(Δt) between the re-addition of extracellular Ca2+ and the peak of the Ca2+ influx response. For each experiment, 150-200 B cells were analyzed with Igor Proanalysis software (Wavemetrics).

### Calcium influx assay

Splenic B cells were labeled with Indo-1 (Molecular Probes) and stained with surface markers to identify each individual subset of B cells. Calcium influx of B cells resuspended in 2×106 cell/ml RPMI 2% FCS was assayed by measurement of 405nm/485nm emission ration after excitation with a 350nm UV laser on a FACS Vantage flow cytometer (BD). Data were analyzed with FlowJo software.

### Somatic hypermutation analysis

The mutational status of the VH186.2 gene was analyzed as described. Briefly, GC (CD38loFashiB220+) and na.ve (CD38+FasloB220+) B-cells were sorted from spleenocytes of wild type or Stim1&2 floxed/floxed, mb1Cre+ mice 7 days after immunization with 100μg of NP-CFF. Genomic DNA from 104 cell equivalents were subjected to two round of genomic PCR amplification protocol using the Expanded High Fidelity PCR system (Roche, Nutley, NJ) and primers previously described G. Esposito et al., Proc Natl Acad Sci U S A 97, 1166 (Feb 1, 2000). PCR fragments corresponding to the Vh186.2 gene were cloned into the pGEM-T easy (Promega) and sequenced using Sanger sequencing. Sequence analysis was performed with the help of DNAStar Lasergene software.

### Statistics

Averages, geometric means, standard deviations, logarithmic standard deviations or medians were calculated depending on the distribution of the data and as indicated. P-values were determined by applying two-tailed Student's T-test for unpaired or paired samples to data sets as appropriate.

## Abbreviations

Stim: STromal Interacting Molecule
ER: Endoplasmic reticulum
BCR: B cell antigen receptor
TCR: T lymphocyte antigen receptors
PIP2: Phosphatidylinositol 4,5 biphophate
IP3: Inositol 1,4,5-triphohphate
CRAC channels: Calcium-Release Activate Calcium Channels
Tregs: T regulatory cells
NFAT: Nuclear factor of activated T cells
GC: Germinal centers
SHM: Somatic hypermutation
FDCs: Follicular dendritic cells
MS: Multiple sclerosis
SOC: Store-Operated Calcium
NP-Ficoll: Nitro-phenylacetyle coupled to Ficoll
TD: T-dependent
TI: T-independent
NP-CGG: 4-hydroxy-3-nitrophenylacetyl chicken γ-globulin
PE: Phecoerythrin
PerCP: Peridin-Chlorophyll
APC: Allophycocyanin
